The article "Insulin Resistance and Biological Aging: The Role of Body Mass, Waist Circumference, and Inflammation" was published in 2022. Journal: Biomed Res Int.

# Insulin Resistance and Biological Aging: The Role of Body Mass, Waist Circumference, and Inflammation

**DOI:** 10.1155/2022/2146596

**Published:** 2022-05-09

**Authors:** Larry A. Tucker

**Affiliations:** College of Life Sciences, Brigham Young University, Provo, Utah 84602, USA

## Abstract

The purpose of this investigation was to evaluate the association between insulin resistance and biological aging in a randomly selected sample of 2,596 U.S. women and men. Another key objective was to examine the extent to which the insulin resistance and biological aging association was influenced by differences in body mass, waist circumference, and systemic inflammation. Biological aging was indexed using the length of leukocyte telomeres. The homeostatic model assessment (HOMA) was employed to index insulin resistance. The body mass index (BMI) was used to represent body mass independent of height. Waist circumference was used to assess abdominal adiposity, and C-reactive protein (CRP) was measured to index body-wide inflammation. Insulin resistance and telomere length were both treated as continuous variables. Results revealed that insulin resistance was related significantly with cellular aging, after adjusting for several demographic covariates (*F* = 5.7, *P* = 0.0234). The association remained significant after controlling for multiple demographic and lifestyle covariates together (*F* = 4.6, *P* = 0.0410). However, after controlling for BMI, along with the other covariates, insulin resistance was no longer associated with biological aging (*F* = 2.1, *P* = 0.1573). After adjusting for differences in waist circumference, along with the demographic and lifestyle covariates, but not BMI, the relationship between insulin resistance and biological aging was negated further (*F* = 1.5, *P* = 0.2283). Adjusting for CRP with the demographic and lifestyle covariates, but not BMI or waist circumference, weakened the relationship (*F* = 4.0, *P* = 0.0552). Evidently, if all adults in the U.S. had the same BMI or waist circumference, there would not be a relationship between insulin resistance and telomere length. It appears that insulin resistance accounts for differences in biological aging mainly because of differences in BMI and waist circumference, especially the latter.

## 1. Introduction

Diabetes mellitus is an important risk factor for many diseases. Research shows that diabetes leads to cardiovascular disease, including coronary heart disease, heart failure, atrial fibrillation, stroke, peripheral artery disease, and other serious disorders [1–3]. Based on NHANES findings in the United States, more than 23 million adults have diagnosed diabetes and almost 8 million more are undiagnosed cases [4]. A staggering 82 million American adults have prediabetes [4].

Type 2 diabetes is generally described as the body's failure to respond to the consumption of a glycemic load with the appropriate amount of insulin to enable glucose uptake [5, 6]. The inability to respond correctly usually happens gradually and is typically a result of insulin resistance. As the disease progresses, insensitivity to insulin leads to elevated blood glucose levels and eventually diabetes [5, 6].

Hyperglycemia causes injury to multiple body systems. Over time, the damage manifests itself in the form of chronic disease and premature mortality. U.S. diabetics have a mortality rate that is roughly 3.5 times the level of nondiabetics [7]. However, before the onset of overt disease and premature death, less obvious health problems can often be detected. For example, insulin resistance leads to chronic inflammation and oxidative stress, important mechanisms of biologic aging [8]. Although less apparent than overt disease, premature biological aging can be evaluated.

A good measure of biological aging is the length of leukocyte telomeres. Telomere length is a meaningful index of cellular senescence [9]. Telomeres are repetitive DNA sequences at the ends of linear chromosomes. They are comprised of proteins and nucleotides of TTAGGG repeats. Although telomeres account for a very small part of the total genomic DNA in a cell, telomeres play a major role in the protection of chromosomes [10]. They cap DNA and help to prevent fusion and injury to the ends of chromosomes. Telomeres gradually shorten with each cell division in the absence of telomerase activity. Although time and number of cell divisions are the best predictors of telomere shortening, many diseases and lifestyle factors also account for differences in telomere length and biological aging [11].

Research indicates that diabetics tend to have shorter telomeres than their counterparts [12, 13], although some research does not support this finding [14]. Similarly, insulin resistance appears to be inversely related to telomere length [15–17]. As insulin resistance increases, telomere length tends to decrease, signifying increased cellular aging.

Obesity also accounts for shorter telomeres, suggesting increased cellular aging, as shown in a meta-analysis by Mundstock et al. [18]. Additionally, abdominal obesity is related significantly with shorter telomeres [19, 20], perhaps even more than elevated BMI levels. Moreover, obesity and abdominal adiposity are closely tied to insulin resistance and diabetes [21, 22]. Clearly, insulin resistance, obesity and central adiposity, and biological aging are closely intertwined.

The significant connection between insulin resistance, obesity, abdominal obesity, and biological aging is thought to be partly the result of systemic inflammation. Many studies have shown that as body-wide inflammation increases, insulin resistance also increases [23]. Similarly, research indicates that there are close ties between obesity and abdominal obesity and systemic inflammation [24].

To date, research has not directly addressed the extent to which the relationship between insulin resistance and biological aging (telomere length) is a result of differences in body mass (BMI), waist circumference, or inflammation. Hence, the present investigation was conducted. This study was designed to determine the extent of the association between insulin resistance and leukocyte telomere length in a large, randomly selected sample of adults, representative of the noninstitutionalized, civilian women and men in the United States. Another objective of the study was to ascertain the extent to which the relationship between insulin resistance and telomere length was a result of differences in body mass (BMI), abdominal adiposity (waist circumference), or systemic inflammation.

## 2. Methods

### 2.1. Study Design

Data from the National Health and Nutrition Examination Survey (NHANES) were used to answer the research questions based on a cross-sectional design. NHANES utilizes a sophisticated, multistage random sampling technique to collect data on thousands of individuals each year, representative of noninstitutionalized civilians living in the United States. The raw data are published online and are free [25]. Data from two consecutive 2-year cycles (NHANES 1999–2000 and 2001–2002) were used in the present investigation. These are the only years that the NHANES collected data on telomere length (biological aging), so data files collected during other years could not be used in this study. The ethics review board of the National Center for Health Statistics approved the NHANES measurement procedures, data collection, and online posting of the data files for public use [26].

### 2.2. Subjects

Participants in the present investigation were 20–84 years old. They represented all regions of the United States and all racial and ethnic groups.

Fasting blood glucose and fasting blood insulin were used to calculate insulin resistance. Therefore, participation in this study required subjects to fast overnight. NHANES did not require all participants to fast, only a 50% subsample of randomly selected adults. Consequently, the total sample for this investigation was 2,596 adults. Participants were each assigned an individual sample weight, so the subsample that fasted was representative of the U.S. adult noninstitutionalized population.

### 2.3. Measures

Insulin resistance, indexed using the homeostatic model assessment (HOMA-IR), was the exposure variable in this study. The outcome variable was the length of leukocyte telomeres, an index of cellular senescence. Age, sex, and race were used as demographic covariates. Pack-years of cigarette smoking, alcohol use, and total physical activity were included as lifestyle covariates. Body mass (BMI) and abdominal adiposity (waist circumference) were the key covariates, employed to determine if the relationship between insulin resistance and biological aging (telomere length) was a result of differences in these potential mediating variables.

#### 2.3.1. Homeostasis Model of Assessment (HOMA-IR)

Insulin resistance is frequently measured using the homeostasis model assessment, commonly known as HOMA-IR. Over 350 research articles have “HOMA” or “HOMA-IR” in their titles, and almost 19,000 scientific articles include “HOMA” or “HOMA-IR” in their reports. HOMA is the most common measure of insulin resistance in the literature.

Development of type 2 diabetes can be accurately predicted using HOMA-IR, independent of body fat distribution, obesity, and glucose tolerance status [27]. Likewise, HOMA-IR is a good predictor of future development of prediabetes among those with normal glucose tolerance [28].

Fasting glucose and fasting insulin levels are used to calculate HOMA-IR. The specific formula employed in the present study was fasting insulin (*μ*U/mL) × fasting plasma glucose (mg/dL)/405. NHANES provides detailed laboratory manuals explaining the procedures used to measure fasting glucose and fasting insulin [29–32].

#### 2.3.2. Leukocyte Telomere Length

Leukocyte telomere length is a good gauge of cell senescence and biological aging [9–11]. According to NHANES, “the telomere length assay was performed in the laboratory of Dr. Elizabeth Blackburn at the University of California, San Francisco, using the quantitative polymerase chain reaction method to measure the telomere length relative to standard reference DNA (T/S ratio), as described in detail elsewhere [33]. Each sample was assayed 3 times on 3 different days. The samples were assayed on duplicate wells, resulting in 6 data points. Sample plates were assayed in groups of 3 plates, and no 2 plates were grouped together more than once. Each assay plate contained 96 control wells with 8 control DNA samples. Assay runs with 8 or more invalid control wells were excluded from further analysis (<1% of runs). Control DNA values were used to normalize between-run variability. Runs with more than 4 control DNA values falling outside 2.5 standard deviations from the mean for all assay runs were excluded from further analysis (<6% of runs). For each sample, any potential outliers were identified and excluded from the calculations (<2% of samples). The mean and standard deviation of the T/S ratio were then calculated normally. The interassay coefficient of variation was 6.5%” [34]. The following formula was used to convert average *T*/*S* ratios to base pairs: 3,274 + 2,413 × (*T*/*S*).

#### 2.3.3. Age

Individuals who were 85 years of age or older were each recorded as 85 years of age by NHANES to maximize confidentiality. Consequently, adults who reported they were 85 or more years old were not included in the study. The minimum age to be a participant was 20 years and the maximum was 84 years.

#### 2.3.4. Race

NHANES categorized adults into 5 racial groups: non-Hispanic White, non-Hispanic Black, Mexican American, other race (including multiracial), and other Hispanic.

#### 2.3.5. Weight

Weight was measured using a digital scale. Subjects wore a standard gown consisting of disposable slippers, pants, and shirt. For participants weighing over 440 pounds, weight was measured using two portable scales. The subject was weighed with one foot on each scale and the two values were summed to estimate total body weight.

#### 2.3.6. Height

A fixed stadiometer with an adjustable headboard was utilized to measure standing height. Subjects were asked to place the back of their head and their heels against the stadiometer. Participants were requested to stand as tall as possible, take a deep breath, and then hold their position until the measurement was completed.

#### 2.3.7. Body Mass Index

Body mass index (BMI) is frequently used to index body weight or mass, independent of height. BMI is calculated by taking weight in kilograms and dividing by height in meters, squared (kg/m^2^). Standard classifications for BMI are as follows: underweight (<18.5), normal weight (18.5–24.99), overweight (25.0–29.99), and obese (≥30.0). BMI was employed as a covariate in this study.

#### 2.3.8. Waist Circumference

Waist circumference is an excellent index of abdominal obesity and central adiposity [35]. Waist circumference was used as a key covariate in the present investigation. According to NHANES, to measure waist circumference, the examiner located the lateral border of the ilium. A horizontal line was drawn using a cosmetic pencil just above the uppermost lateral border of the right ilium. A vertical line was then drawn marking the midaxillary line. A steel measuring tape was extended around the waist at the level of the superior lateral border of the iliac crests, with the examiner making sure that the tape stayed horizontal and parallel to the floor. The measurement was not to compress the skin, but the tape was to be snug. The waist measurement was taken to the nearest 0.1 cm after the subject exhaled one normal breath [36].

#### 2.3.9. Smoking

Cigarette smoking was used as a covariate. Specifically, pack-years of smoking were used to estimate the long-term use of cigarettes. Pack-years were calculated by multiplying the number of packs of cigarettes smoked per day by the number of years the person reported smoking. A pack of cigarettes was defined as 20 cigarettes.

#### 2.3.10. Alcohol Use

NHANES used three categories to account for differences in alcohol consumption: abstainers, moderate drinkers, and heavy drinkers. Abstainers were adults who reported that they did not drink alcohol. Moderate drinkers were men who reported that they drank >0 and <3 drinks per day or women who indicated that they drank >0 and <2 drinks per day. Heavy drinkers were men who reported that they consumed 3 or more alcoholic drinks per day or women who reported that they drank 2 or more drinks per day. Alcohol use was employed as a covariate in this study.

#### 2.3.11. Total Physical Activity

MET minutes were used to index total physical activity. A MET is a metabolic equivalent, the amount of energy expended at rest. Casual walking produces about three METs, triple the energy expenditure compared to sitting. If a person engaged in casual walking for 30 minutes, then, MET minutes would be 90 (3 METs × 30 minutes). Participants were asked to report which, if any, of a list of 48 physical activities they engaged in during the past 30 days. Choices included activities such as tennis, walking, gardening, hiking, swimming, bicycling, and 42 others. Subjects reported if the intensity of each activity that they engaged in was moderate or vigorous using NHANES definitions. Using the compendium of physical activity, a MET value for each activity was assigned [37]. By summing the MET minutes of each activity and converting the score to a weekly value, a total physical activity score was calculated and used as a covariate.

#### 2.3.12. Systemic Inflammation

Blood levels of C-reactive protein (CRP) were measured to index systemic inflammation. CRP is considered one of the best measures of systemic inflammation. Latex-enhanced nephelometry was utilized to quantify CRP levels (mg/dL). According to NHANES [38], particle-enhanced assays were based on the reaction between a soluble analyte and the corresponding antigen or antibody bound to polystyrene particles. For the quantification of CRP, particles consisting of a polystyrene core and a hydrophilic shell were used to link anti-CRP antibodies covalently. A dilute solution of the test sample was mixed with latex particles coated with mouse monoclonal anti-CRP antibodies. CRP present in the test sample formed an antigen-antibody complex with the latex particles. An automatic blank subtraction was then performed. CRP concentrations were calculated by using a calibration curve. Data reduction of the signals was performed by using a storable logit-log function for the calibration curve. The assays were completed on a Behring nephelometer for quantitative CRP determination, according to the laboratory methodology described by the NHANES [38].

### 2.4. Data Analysis

NHANES participants were randomly selected using a multilevel, probability, sampling strategy. A total of 28 strata and 57 clusters were randomly selected. Additionally, NHANES assigned each subject an individual sample weight. Because the sample weights were used as part of each analysis, unbiased national estimates resulted. In short, the findings can be generalized to the noninstitutionalized, civilian adult population in the United States. Because of nesting, each analysis was based on 29 degrees of freedom (df) in the denominator (57 clusters minus 28 strata). Statistical significance was based on the 29 df, not the 2,596 subjects in the study.

Continuous variables were summarized using means (±SE) and categorical variables were described using frequencies (±SE). Regression analysis using the SAS SURVEYREG procedure was employed to determine the extent of the linear association between insulin resistance and telomere length, each treated as a continuous variable. Regression coefficients were reported showing the extent to which telomere lengths varied based on differences in HOMA-IR. Partial correlation was used to adjust for differences in the covariates, specifically, age, sex, race, smoking, alcohol use, total physical activity, BMI, waist circumference, and CRP. The SAS variance inflation factor (VIF) was used to determine the extent of multicollinearity in the regression models.

SAS version 9.4 (SAS Institute Inc., Cary, NC) was the software run to conduct the statistical analyses. All *P* values were two sided, and statistical significance was accepted when alpha was less than 0.05.

## 3. Results

A total of 1,310 women and 1,286 men, representative of the U.S. adult population, were included in the analyses. The mean age (±SE) was 46.4 (±0.8) years. The average telomere length in base pairs and HOMA-IR were 5812.5 (±50.6) and 3.3 (±0.07), respectively. The mean BMI and waist circumference (cm) were 28.3 (±0.18) and 96.8 cm (±0.37), respectively. The mean CRP was 0.43 (±0.03).  Table 1 shows a summary of the percentiles (±SE) for the continuous variables of the investigation.

Across the sample, chronological age was linearly associated with the length of leukocyte telomeres (*r* = 0.41, *P* < 0.0001). There was not a quadratic relationship between age-squared and telomere lengths beyond the linear association (*F* = 2.8, *P* = 0.1067). In the present study, telomeres were 16.8 base pairs shorter for each year of chronological age (*F* = 120.4, *P* < 0.0001).

Treating both insulin resistance (HOMA-IR) and telomere length as continuous variables revealed a significant linear association between the exposure and outcome variables with 29 df, as displayed in Table 2. Controlling only for the demographic covariates (age, sex, and race) resulted in a significant relationship (*F* = 5.7, *P* = 0.0234). Likewise, after adding the lifestyle covariates (pack-years of smoking, total physical activity, and alcohol use) to the demographic covariates, the association between HOMA-IR and telomere length remained significant (*F* = 4.6, *P* = 0.0410). However, adjusting for differences in BMI, along with the demographic and lifestyle covariates, weakened the relationship and it was no longer statistically significant (*F* = 2.1, *P* = 0.1573). Controlling for differences in waist circumference instead of BMI, along with the demographic and lifestyle covariates, attenuated the association more, and the connection between insulin resistance and telomere length was further nullified (*F* = 1.5, *P* = 0.2283). Multicollinearity was not a threat in any of these models. In all cases, the variance inflation factor (VIF) remained minimal (<1.5).

The relationship between BMI and CRP was significant with age, sex, and race controlled (*F* = 54.0, *P* < 0.0001). For each 10-unit increase in BMI, CRP increased by 0.3 mg/dL. Similarly, the association between waist circumference and CRP was significant after controlling for the same covariates (*F* = 56.7, *P* < 0.0001). For each 10 cm increase in waist circumference, CRP increased by 0.1 mg/dL. The difference between CRP scores representing the 5th percentile of the U.S. population to the 50th percentile was about 0.2 mg/dL. With age, sex, race, smoking, physical activity, and alcohol use controlled, CRP was related significantly to telomere length (*F* = 6.9, *P* = 0.0138). Specifically, for each 1 mg/dL increase in CRP, telomeres were 52 base pairs shorter. Adjusting for differences in systemic inflammation (C-reactive protein), along with all the other covariates, except BMI or waist circumference, weakened the relationship between HOMA-IR and telomere length to the point of borderline significance (*F* = 4.0, *P* = 0.0552).

## 4. Discussion

The present investigation had three primary objectives. The first aim was to determine the relationship between insulin resistance and biological aging in a large, randomly selected sample of women and men representative of the U.S. adult population. The second purpose was to ascertain the extent to which the insulin resistance and telomere length association was affected by body mass (BMI) and/or abdominal adiposity (waist circumference). The third objective was to evaluate the relationship between insulin resistance and telomere length with systemic inflammation controlled, along with age, sex, race, smoking, total physical activity, and alcohol use.

Findings revealed that the association between insulin resistance, measured by HOMA-IR, and biological aging, indexed using leukocyte telomere length, was linear, significant, and meaningful. The relationship remained linear, significant, and meaningful after adjusting for differences in age, sex, and race and also after controlling for total physical activity, alcohol use, and smoking pack-years, in addition to the demographic factors. However, the association was nullified after controlling statistically for differences in BMI and was weakened further after adjusting for differences in waist circumference, instead of BMI. In short, the results indicated that body mass and waist circumference each individually mediated the relationship between insulin resistance and telomere length. Stated another way, if all U.S. adults had the same BMI or if they all had the same waist size, there would not be an association between insulin resistance and biological aging.

Adjusting for differences in CRP with the other covariates, except BMI or waist circumference, also weakened the insulin resistance and telomere length relationship, but the association remained borderline significant. Apparently, the length of telomeres tends to be shorter as insulin resistance increases, mostly because adults who are insulin resistant tend to be more overweight or obese or they tend to have more abdominal adiposity than their counterparts. Systemic inflammation seems to also play a role, but the role of inflammation appears less important than the role of BMI and abdominal adiposity.

In the present study, after adjusting for differences in the demographic and lifestyle covariates, telomere length was 10.7 base pairs shorter for each one-unit increase in HOMA-IR. Additionally, multiple regression analysis showed that a difference of 16.8 base pairs was equal to one year of chronological aging. Hence, the difference between adults 40 years old and those aged 70 would be roughly 504 telomere base pairs, on average, or 30 years of aging (30 × 16.8 = 504).

In the present study, the 25th percentile for HOMA-IR was 1.5 ± 0.0 and the 75th percentile was 3.8 ± 0.1 (see Table 1), a difference of 2.3 HOMA-IR units. Therefore, the estimated cellular aging difference between adults at the 25th percentile and those at the 75th percentile was approximately 24.6 telomere base pairs (2.3 × 10.7 = 24.6). Hence, the biologic aging difference between adults at the HOMA-IR 25th and 75th percentiles was approximately 2.3 years (24.6 ÷ 10.7 = 2.3).

Other studies have calculated the biological aging difference between groups based on various lifestyle factors. For example, U.S. adults reporting 25 smoking pack-years have about 4.6 years of advanced cellular aging compared to nonsmokers [39]. Similarly, for each serving of sugar-sweetened soda consumed per day, telomeres tend to be 1.8 years shorter, on average [40]. Finally, adults who eat nuts and seeds regularly tend to have telomeres that are longer by 1.7 years, on average, compared to their counterparts [41].

A number of studies have shown that insulin resistance and telomere length are related significantly. However, few if any investigations, to date, have shown that the relationship between insulin resistance and telomere length is mediated by body mass and central adiposity. For example, in a study by Adaikalakoteswari et al. [17], 40 type II diabetics were compared to 40 age- and sex-matched controls. Results showed that insulin resistance (HOMA-IR) was related significantly to terminal restriction fragment (*r* = −0.4, *P* = 0.01), a measure of average telomere length. Differences in abdominal adiposity and/or BMI were not controlled, however.

Demissie et al. [16] studied insulin resistance and leukocyte telomere length in 327 Caucasian men from the Framingham Heart Study. Terminal restriction fragment (TRF) length was employed to index telomere length. TRF was correlated weakly with HOMA-IR (*r* = −0.16, *P* = 0.007), but the mediating role of waist size and/or BMI was not evaluated. Similarly, cross-sectional research by Al-Attas et al. [42] using 193 adults indicated that HOMA-IR and LTL were associated significantly (*r* = −0.29, *P* < 0.01) but neither BMI nor waist size was controlled. Furthermore, chronological age was not related to telomere length (*r* = 0.00, *P* > 0.5), even though age range of the sample was 18–66 years.

In an investigation by Strazhesko et al. [15], the relationship between HOMA-IR and telomere length was studied in 274 subjects with a wide age range, 23–91 years. Specific correlation coefficients were not given, but the HOMA and telomere association was deemed significant (*P* < 0.0001). As with the other investigations, the mediating effects of abdominal adiposity and BMI on the insulin resistance and telomere length relationship were not reported.

Finally, Wang et al. [43] conducted a meta-analysis using 17 studies that investigated the association between diabetes and telomere length. Although there were major differences between the present study, which focused on insulin resistance in nondiabetics, and the meta-analysis, which focused on diabetics, general parameters were similar. Findings showed that diabetics had shorter telomeres than nondiabetics, although a publication bias was noted. Although BMI was not controlled statistically, studies were separated based on categories of BMI, allowing effect modification to be evaluated. Results indicated that the relationship between diabetes status and telomere length was weaker in the obese compared to the other BMI categories, suggesting that obesity plays a role in the association.

There are several interrelated mechanisms that could account for the outcomes of this investigation. Research indicates that obesity, insulin resistance, oxidative stress, inflammation, and cell aging are interconnected [43, 44]. In the present study, BMI and abdominal obesity were both strongly related to systemic inflammation (CRP) and CRP was strongly related to biological aging. Without differences in obesity and/or abdominal obesity and to a lesser extent systemic inflammation, the connection between insulin resistance and biological aging appears to be minimal.

Immune system responses to bodily insults result in inflammation [45]. In many ways, obesity acts as an insult to the body [23]. The literature is filled with research showing that obesity and abdominal adiposity promote increased levels of inflammation [24]. Similarly, there is a plethora of studies connecting insulin resistance with obesity and inflammation [23, 46]. The literature also shows that reactive oxygen species (ROS) contribute significantly to the inflammatory processes [47]. In short, chronic inflammation and oxidative stress are strongly interconnected. Therefore, it follows that oxidative stress also plays an important part in biological aging [48].

Evidence suggests that oxidative stress leads to shortened telomeres [49]. Research by von Zglinicki [50] and others reviewed by Houben et al. [48] using a variety of animal species support this relationship. Since adults with obesity are inclined to have increased oxidative stress and chronic inflammation [51, 52], it follows that these individuals would also tend to have shorter telomeres [49, 50].

Obesity leads to inflammatory cytokine activation with increased markers of fatty acid-induced oxidative and endoplasmic reticulum stress in a variety of tissues [43, 53]. Obesity also causes insulin resistance and beta-cell apoptosis [54]. Insulin resistance typically precedes the onset of type II diabetes. Moreover, oxidative stress appears to be a meaningful predictor of the development of insulin resistance later in life [55]. Finally, because telomeres have high levels of guanine, one of the four bases of nucleic acids, and guanine is especially vulnerable to oxidative stress, telomeres tend to be damaged by obesity, insulin resistance, and diabetes [56]. Other factors, such as oxidative stress associated with mitochondrial injury and nuclear somatic mutations, also contribute to biological aging [57].

More than 90% of type 2 diabetics are overweight or obese [58]. Clearly, obesity plays a key role in the oxidative stress, beta-cell injury, insulin resistance, diabetes, and telomere attrition cascade. Given that the results of the present study show that the association between insulin resistance and telomere length collapses when adjustments are made for differences in body mass or abdominal adiposity, it appears that they are the likely drivers of the relationship.

The present investigation was not without limitations. First, because the study was based on a cross-sectional design, cause-and-effect conclusions are not warranted. Second, adults with insulin resistance may be an exclusive group of individuals with unique lifestyles and characteristics. In the present study, many covariates were controlled statistically to minimize this threat but there are always unidentified variables that could account for the association between insulin resistance and biological aging and the mediating influence of obesity.

This investigation also had several strengths. First, subjects were randomly selected from all noninstitutionalized, civilian adults in the U.S. 20–84 years of age. Hence, the findings can be generalized broadly. Second, high-quality, objective measurement methods were employed to assess the outcome and exposure variables. Third, all the variables were measured by well-trained, independent scientists, unrelated to the present study, so there were no experimenter biases affecting data collection. Fourth, a large sample was studied, approximately 2,600 participants, so outcomes were stable. Fifth, the relationship between age and telomere length was linear and significant, as it should be, adding credence to the telomere measurement process.

## 5. Conclusion

In conclusion, as insulin resistance increases in U.S. adults, cellular aging increases linearly. However, after controlling for BMI and/or waist circumference, there is no relationship between insulin resistance and telomere length. Evidently, if adults in the U.S. all had the same level of body mass or waist size, there would not be a relationship between insulin resistance and biological aging. It appears that the association between insulin resistance and cellular aging is partly a function of differences in body mass, especially abdominal adiposity.

## Figures and Tables

**Table 1:** Percentiles for the key continuous variables representing U.S. women and men.

Variable	Percentile (±SE)				
	5th	25th	50th	75th	95th
HOMA-IR	1.0 ± 0.0	1.5 ± 0.0	2.4 ± 0.0	3.8 ± 0.1	8.5 ± 0.4
Smoking (pack-years)	0.0 ± 0.2	0.0 ± 0.2	0.0 ± 0.2	0.0 ± 0.2	22.4 ± 2.6
Age (years)	21.7 ± 0.4	33.3 ± 1.0	44.2 ± 1.1	57.7 ± 1.2	75.1 ± 1.2
Body mass index (kg/m^2^)	20.1 ± 0.1	24.0 ± 0.2	27.2 ± 0.1	31.3 ± 0.3	40.3 ± 0.8
Total activity (MET minutes)	0.0 ± 4	0.0 ± 4	0.0 ± 4	138.8 ± 17	508.0 ± 33
Waist circumference (cm)	73.5 ± 0.5	85.7 ± 0.6	95.7 ± 0.4	105.9 ± 0.4	124.7 ± 1.7
C-reactive protein (mg/dL)	0.02 ± 0.00	0.09 ± 0.00	0.21 ± 0.01	0.46 ± 0.02	1.58 ± 0.10
Telomere length (base pairs)	4,921 ± 36	5,365 ± 46	5,717 ± 43	6,140 ± 51	7,022 ± 124

SE: standard error. Table values include person-level weighted adjustments based on the sampling methods of NHANES so that values represent those of the U.S. adult population.

**Table 2:** Relationship between HOMA-IR and telomere length (base pairs) in U.S. women and men, after adjusting for the covariates.

Exposure variable	Telomere length (base pairs)			
	Regression coefficient	SE	*F*	*P*
HOMA-IR				
Model 1	−10.4	4.4	5.7	0.0234
Model 2	−10.7	5.0	4.6	0.0410
Model 3	−6.6	4.6	2.1	0.1573
Model 4	−6.6	5.4	1.5	0.2283
Model 5	−9.3	4.7	4.0	0.0552

SE: standard error of the regression coefficient. For model 1, the covariates were age, sex, and race. For model 2, in addition to age, sex, and race, the model was adjusted for differences in pack-years of smoking, alcohol use, and total physical activity. Model 3 included the same covariates as model 2 but also included BMI. Model 4 included the same covariates as model 2 but also included waist circumference. Model 5 included the same covariates as model 2 but also included CRP. Interpretation of the regression coefficients is as follows for the first row (model 1) regarding HOMA-IR and telomere length with age, sex, and race controlled statistically: for each one-unit increase in HOMA-IR, telomeres were 10.4 base pairs shorter, on average, signifying increased biological aging.

## Data Availability

All data used in the present study are available online as part of the National Health and Nutrition Examination Survey (NHANES). The data are free and can be accessed by using the following Centers for Disease Control and Prevention website: https://wwwn.cdc.gov/nchs/nhanes/Default.aspx

## References

[1] Yu M., Zhang X., Lu F., Fang L. (2015). Depression and risk for diabetes: a meta-analysis. *Canadian Journal of Diabetes*.

[2] Pop-Busui R., Boulton A. J., Feldman E. L. (2017). Diabetic neuropathy: a position statement by the American Diabetes Association. *Diabetes Care*.

[3] Das R. N. (2016). Relationship between diabetes mellitus and coronary heart disease. *Current Diabetes Reviews*.

[4] Benjamin E. J., Virani S. S., Callaway C. W. (2018). Heart Disease and Stroke Statistics-2018 update: a report from the American Heart Association. *Circulation*.

[5] DeFronzo R. A. (2004). Pathogenesis of type 2 diabetes mellitus. *The Medical Clinics of North America*.

[6] Stumvoll M., Goldstein B. J., van Haeften T. W. (2005). Type 2 diabetes: principles of pathogenesis and therapy. *Lancet*.

[7] Stokes A., Mehta N. K. (2013). Mortality and excess risk in US adults with pre-diabetes and diabetes: a comparison of two nationally representative cohorts, 1988-2006. *Population Health Metrics*.

[8] Jha J. C., Ho F., Dan C., Jandeleit-Dahm K. (2018). A causal link between oxidative stress and inflammation in cardiovascular and renal complications of diabetes. *Clinical Science (London, England)*.

[9] Bernadotte A., Mikhelson V. M., Spivak I. M. (2016). *Markers of Cellular Senescence. Telomere Shortening as a Marker of Cellular Senescence*.

[10] Shay J. W. (2018). Telomeres and aging. *Current Opinion in Cell Biology*.

[11] Blasco M. A. (2005). Telomeres and human disease: ageing, cancer and beyond. *Nature Reviews. Genetics*.

[12] Zee R. Y., Castonguay A. J., Barton N. S., Germer S., Martin M. (2010). Mean leukocyte telomere length shortening and type 2 diabetes mellitus: a case-control study. *Translational Research*.

[13] Zhao J., Miao K., Wang H., Ding H., Wang D. W. (2013). Association between telomere length and type 2 diabetes mellitus: a meta-analysis. *PLoS One*.

[14] Menke A., Casagrande S., Cowie C. C. (2015). Leukocyte telomere length and diabetes status, duration, and control: the 1999-2002 National Health and Nutrition Examination Survey. *BMC Endocrine Disorders*.

[15] Strazhesko I., Tkacheva O., Boytsov S. (2015). Association of insulin resistance, arterial stiffness and telomere length in adults free of cardiovascular diseases. *PLoS One*.

[16] Demissie S., Levy D., Benjamin E. J. (2006). Insulin resistance, oxidative stress, hypertension, and leukocyte telomere length in men from the Framingham Heart Study. *Aging Cell*.

[17] Adaikalakoteswari A., Balasubramanyam M., Ravikumar R., Deepa R., Mohan V. (2007). Association of telomere shortening with impaired glucose tolerance and diabetic macroangiopathy. *Atherosclerosis*.

[18] Mundstock E., Sarria E. E., Zatti H. (2015). Effect of obesity on telomere length: systematic review and meta-analysis. *Obesity (Silver Spring)*.

[19] Mangge H., Renner W., Almer G. (2019). Subcutaneous adipose tissue distribution and telomere length. *Clinical Chemistry and Laboratory Medicine*.

[20] Lee M., Martin H., Firpo M. A., Demerath E. W. (2011). Inverse association between adiposity and telomere length: the Fels Longitudinal Study. *American Journal of Human Biology*.

[21] Firouzi S. A., Tucker L. A., LeCheminant J. D., Bailey B. W. (2018). Sagittal abdominal diameter, waist circumference, and BMI as predictors of multiple measures of glucose metabolism: an NHANES investigation of US adults. *Journal Diabetes Research*.

[22] Nordfjall K., Eliasson M., Stegmayr B., Lundin S., Roos G., Nilsson P. M. (2008). Increased abdominal obesity, adverse psychosocial factors and shorter telomere length in subjects reporting early ageing; the MONICA Northern Sweden Study. *Scandinavian Journal of Public Health*.

[23] Wu H., Ballantyne C. M. (2020). Metabolic inflammation and insulin resistance in obesity. *Circulation Research*.

[24] Karczewski J., Sledzinska E., Baturo A. (2018). Obesity and inflammation. *European Cytokine Network*.

[25] NHANES Data Files: Questionnaires, Datasets, and Related Documentation. https://wwwn.cdc.gov/nchs/nhanes/Default.aspx.

[26] NHANES Research Ethics Review Board (ERB) Approval. https://www.cdc.gov/nchs/nhanes/irba98.htm.

[27] Haffner S. M., Kennedy E., Gonzalez C., Stern M. P., Miettinen H. (1996). A prospective analysis of the HOMA model. The Mexico City Diabetes Study. *Diabetes Care*.

[28] Onishi Y., Hayashi T., Sato K. K. (2010). Fasting tests of insulin secretion and sensitivity predict future prediabetes in Japanese with normal glucose tolerance. *J Diabetes Investig*.

[29] NHANES Labratory Procedure Manual: Serum Insulin. https://wwwn.cdc.gov/nchs/data/nhanes/1999-2000/labmethods/lab10am_met_insulin.pdf.

[30] NHANES Laboratory Procedure Manual: Serum Glucose. https://wwwn.cdc.gov/nchs/data/nhanes/1999-2000/labmethods/lab10am_met_plasma_glucose.pdf.

[31] NHANES Labratory Procedure Manual: Serum Insulin. https://wwwn.cdc.gov/nchs/data/nhanes/2001-2002/labmethods/l10am_b_met_insulin.pdf.

[32] NHANES Laboratory Procedure Manual: Plasma Glucose. https://wwwn.cdc.gov/nchs/data/nhanes/2001-2002/labmethods/l10am_b_met_glucose.pdf.

[33] Needham B. L., Adler N., Gregorich S. (2013). Socioeconomic status, health behavior, and leukocyte telomere length in the National Health and Nutrition Examination Survey, 1999-2002. *Social Science & Medicine*.

[34] NHANES 2001-2002 Data Documentation, Codebook, and Frequencies. Telomere Mean and Standard Deviation. https://wwwn.cdc.gov/Nchs/Nhanes/2001-2002/TELO_B.htm.

[35] Ross R., Leger L., Morris D., de Guise J., Guardo R. (1992). Quantification of adipose tissue by MRI: relationship with anthropometric variables. *Journal of Applied Physiology*.

[36] NHANES Anthropometry Procedures Manual. https://wwwn.cdc.gov/nchs/data/nhanes/2017-2018/manuals/2017_Anthropometry_Procedures_Manual.pdf.

[37] Ainsworth B. E., Haskell W. L., Whitt M. C. (2000). Compendium of physical activities: an update of activity codes and MET intensities. *Medicine and Science in Sports and Exercise*.

[38] NHANES C-Reactive protein (CRP), Fibrinogen, Bone Alkaline Phosphatase & Urinary N-telopeptides. https://wwwn.cdc.gov/Nchs/Nhanes/2001-2002/L11_B.htm.

[39] Tucker L. A. (2017). Caffeine consumption and telomere length in men and women of the National Health and Nutrition Examination Survey (NHANES). *Nutrition & Metabolism (London)*.

[40] Leung C. W., Laraia B. A., Needham B. L. (2014). Soda and cell aging: associations between sugar-sweetened beverage consumption and leukocyte telomere length in healthy adults from the National Health and Nutrition Examination Surveys. *American Journal of Public Health*.

[41] Tucker L. A. (2017). Consumption of nuts and seeds and telomere length in 5,582 men and women of the National Health and Nutrition Examination Survey (NHANES). *The Journal of Nutrition, Health & Aging*.

[42] Al-Attas O. S., Al-Daghri N. M., Alokail M. S. (2010). Adiposity and insulin resistance correlate with telomere length in middle-aged Arabs: the influence of circulating adiponectin. *European Journal of Endocrinology*.

[43] Wang J., Dong X., Cao L. (2016). Association between telomere length and diabetes mellitus: a meta-analysis. *The Journal of International Medical Research*.

[44] Yang Y., Liu J. L., Hu P. (2013). Association of shortened telomere length with oxidative stress in leukocytes of T1DM and T2DM patients. *Chin Journal of Diabetes*.

[45] Mittal M., Siddiqui M. R., Tran K., Reddy S. P., Malik A. B. (2014). Reactive oxygen species in inflammation and tissue injury. *Antioxidants & Redox Signaling*.

[46] Ying W., Fu W., Lee Y. S., Olefsky J. M. (2020). The role of macrophages in obesity-associated islet inflammation and *β*-cell abnormalities. *Nature Reviews. Endocrinology*.

[47] Fernandez-Sanchez A., Madrigal-Santillan E., Bautista M. (2011). Inflammation, oxidative stress, and obesity. *International Journal of Molecular Sciences*.

[48] Houben J. M., Moonen H. J., van Schooten F. J., Hageman G. J. (2008). Telomere length assessment: biomarker of chronic oxidative stress?. *Free Radical Biology & Medicine*.

[49] Kawanishi S., Oikawa S. (2004). Mechanism of telomere shortening by oxidative stress. *Annals of the New York Academy of Sciences*.

[50] von Zglinicki T. (2002). Oxidative stress shortens telomeres. *Trends in Biochemical Sciences*.

[51] Sarparanta J., Garcia-Macia M., Singh R. (2017). Autophagy and mitochondria in obesity and type 2 diabetes. *Current Diabetes Reviews*.

[52] Boles A., Kandimalla R., Reddy P. H. (2017). Dynamics of diabetes and obesity: epidemiological perspective. *Biochimica et Biophysica Acta - Molecular Basis of Disease*.

[53] (1997). Report of the expert committee on the diagnosis and classification of diabetes mellitus. *Diabetes Care*.

[54] Jonas J. C., Bensellam M., Duprez J., Elouil H., Guiot Y., Pascal S. M. (2009). Glucose regulation of islet stress responses and *β*-cell failure in type 2 diabetes. *Diabetes, Obesity & Metabolism*.

[55] Sampson M. J., Winterbone M. S., Hughes J. C., Dozio N., Hughes D. A. (2006). Monocyte telomere shortening and oxidative DNA damage in type 2 diabetes. *Diabetes Care*.

[56] Ma D., Zhu W., Hu S., Yu X., Yang Y. (2013). Association between oxidative stress and telomere length in type 1 and type 2 diabetic patients. *Journal of Endocrinological Investigation*.

[57] Sozou P. D., Kirkwood T. B. (2001). A stochastic model of cell replicative senescence based on telomere shortening, oxidative stress, and somatic mutations in nuclear and mitochondrial DNA. *Journal of Theoretical Biology*.

[58] Bramante C. T., Lee C. J., Gudzune K. A. (2017). Treatment of obesity in patients with diabetes. *Diabetes Spectrum: A Publication of the American Diabetes Association*.

